The article "Integrated Analysis of DNA Repair Genes Identifies SLC6A1 as a New Marker for the Clinical Outcome of Patients with Colorectal Cancer" was retracted in 2023. Reasons: unreliable results or conclusions; concerns about the data; concerns about the results or conclusions; concerns about the peer review.

# Integrated Analysis of DNA Repair Genes Identifies SLC6A1 as a New Marker for the Clinical Outcome of Patients with Colorectal Cancer

**DOI:** 10.1155/2022/4952812

**Published:** 2022-02-22

**Authors:** Qian-qian Wang, Yang Wei, Li-ping Luo, Xin Li, Wen-jun Jiang

**Affiliations:** ^1^School of Medicine, University of Electronic Science and Technology of China, Chengdu 611731, China; ^2^Department of Medical Oncology, Sichuan Cancer Hospital & Institute, Sichuan Cancer Center, School of Medicine, University of Electronic Science and Technology of China, Chengdu, Sichuan 610041, China; ^3^Radiation Oncology Key Laboratory of Sichuan Province, Sichuan Cancer Hospital & Institute, Sichuan Cancer Center, School of Medicine, University of Electronic Science and Technology of China, Chengdu, Sichuan 610041, China

## Abstract

Colorectal cancer (CRC) remains an important malignancy worldwide with poor prognosis. It has been known that DNA repair genes are involved in the development and progression of various tumors. Therefore, the purpose of this study was to explore DNA repair gene-based prognostic biomarkers for CRC. In this study, the expressing pattern and prognostic values of DNA repair genes in CRC patients were analyzed using TCGA database. GO and KEGG enrichment analyses were conducted to clarify the functional roles of dysregulated genes. We observed 358 differentially expressed DNA repair genes in CRC specimens, including 84 downregulated genes and 275 upregulated genes. 36 survival-related DNA repair genes were correlated with CRC patients' five-year survival, including 6 low-risk genes and 30 high-risk genes. Among the 10 overlapping genes, we focused on SLC6A1 which was highly expressed in CRC, and multivariate analysis confirmed that SLC6A1 expression as well as age and clinical stage could be regarded as an independent predicting factor for CRC prognosis. KEGG assays revealed that SLC6A1 may influence the clinical progression via regulating TGF-beta and PI3K-Akt signaling pathways. In addition, we observed that SLC6A1 was negatively regulated by SLC6A1 methylation, leading to its low expression in CRC specimens. Overall, SLC6A1 is upexpressed in CRC and can be used as a marker of poor prognosis in CRC patients.

## 1. Introduction

Colorectal cancer (CRC), as the third most common cancer in males and second most common in females, affects appropriately 1.85 million people worldwide and accounts for 9.2% of all cancer deaths [1, 2]. CRC is considered to be the leading cause of cancer-related deaths and poses a serious threat to global public health [3, 4]. Although recent developments in colonoscopy have improved outcomes for patients with CRC, 5-year relative survival remains below 50% in low-income countries. Tumor metastasis is the main cause of death in patients with CRC, and patients with metastatic CRC have a poor prognosis [5, 6]. Thus, it is necessary to further explore the mechanism of the CRC progression and recognize reliable diagnostic markers and therapeutic targets for CRC.

As a crucial hallmark of cancer, genomic instability contributes to cancer transformation [7]. Several circulating markers have been shown to possess the ability of predicting treatment response and survival in cancer patients [8, 9]. According to the report, serum lncRNA DANCR expression was distinctly increased in colorectal cancer, and its diagnostic and prognostic values were also demonstrated in CRC patients from both several cohorts [10]. Elevated serum pentraxin-3 level in patients with CRC after therapeutic surgery predicts poor prognosis [11]. Therefore, learning the genetic and epigenetic changes associated with the progression of CRC is a critical issue in providing new therapeutic targets for CRC. Cells have developed a variety of complex DNA repair mechanisms to repair DNA damage, such as DNA damage response (DDR), in order to maintain genomic integrity [12]. DNA repair continues to play a role in human cells to identify and correct damage to the DNA molecules that encode their genomes [13]. Disruption of the DDR process is closely related to the failure of accurate repair of damaged DNA in cells, leading to the transformation of normal cells into tumor cells and the accumulation of genetic changes [14, 15]. In recent years, the use of DNA repair genes (DRGs) as diagnostic or prognostic molecular biomarkers has been paid much attention to by the oncology field [16, 17]. However, the prognostic role of DRGs and their biological function in CRC remained rudimentary and inconclusive.

In this research, we explored DNA repair genes associated with long-term survivals in CRC. Then, our attention focused on SLC6A1 which may be a novel prognostic biomarker for CRC. Moreover, we analyzed the mechanisms involved in the dysregulation of SLC6A1. In general, our findings offered new clues for identifying new biomarkers.

## 2. Materials and Methods

### 2.1. Study Population

In this study, all subjects came from The Cancer Genome Atlas (TCGA), and there were a total of 521 samples, including 480 CRC tumor tissues and 41 adjacent normal tissues.

### 2.2. Differentially Expressed DNA Repair Genes

Data analysis of differentially expressed DNA repair genes between CRC and nontumor specimens was carried out by using package limma in R, and the threshold of |log2 fold change (FC)| was larger than 2, and the adjusted *P* value is less than 0.05 [18]. The expressing patterns of DNA repair genes were demonstrated by volcanic and heat maps.

### 2.3. COX Regression Analysis

Univariate COX regression was used to load the software package lifetime by using R language. We showed the top 40 genes in univariate COX in an ascending order of *P* value. The effects of the SLC6A1 expression and other clinical characteristics (age, sex, and stage) on survival were compared by multivariate Cox analysis. The median value determined the cut-off value of the SLC6A1 expression. If *P* value was less than 0.05, it would be thought significant in all tests.

### 2.4. Functional Enrichment Analysis

GO annotation and KEGG pathway analysis with the clusterProfiler package in R were performed for abnormally expressed genes between CRC specimens with high and low SLC6A1 expression, and *P* value <0.05 was used as the cut-off point for functional pathway evaluation [19].

### 2.5. Correlation Analysis of SLC6A1 mRNA Expression and Methylation of CpG Sites

The Pearson correlation test was used to analyze the correlation between SLC6A1 mRNA expression and CpG methylation in different regions of SLC6A1 gene. The correlation between SLC6A1 mRNA expression and methylation at each CpG site was detected, and *P* < 0.05 was considered to be statistically significant.

### 2.6. Statistical Analysis

The statistical analysis was completed using R program 3.6.1. Student's *t*-test was used to analyze the comparisons between the two independent groups. The Kaplan-Meier method was used to evaluate the overall survival rate of each group, and log-rank test was used to evaluate the differences between groups. *P* < 0.05 was considered to be statistically significant.

## 3. Results

### 3.1. Identification of Differentially Expressed DNA Repair Genes

To identify DNA repair genes involved in the CRC progression, we downloaded a gene list containing 1547 DNA repair genes from GSEA (http://www.gsea-msigdb.org/gsea/index.jsp).Then, we performed “limma” using TCGA datasets and found 358 differentially expressed DNA repair genes in CRC specimens, including 84 downregulated genes and 275 upregulated genes (Figure 1(a) and Supplementary Table S1). In addition, heat map exhibited the expressing pattern of the differentially expressed DNA repair genes in CRC specimens (Figure 1(b)).

### 3.2. The Screen of Survival-Related DNA Repair Genes

Later, univariate analyses were performed to screen for DNA repair genes associated with survival, with the standard of *P* < 0.001. As shown in Figure 2, we found that 36 survival-related DNA repair genes were correlated with CRC patients' five-year survival, including 6 low-risk genes and 30 high-risk genes.

### 3.3. The Identification of Dysregulated and Survival-Related DNA Repair Genes in CRC

To further screen dysregulated and survival-related DNA repair genes in CRC, we performed Venn analysis and identified 10 genes associated with CRC prognosis (Figure 3(a)). Their expressing pattern is exhibited in Figure 3(b) using heat map. The *P* and HR values of the selected 10 genes are shown in Figure 3(c) based on the univariate assays. Moreover, the correlation network results revealed that the expression of SNAI1, TCF7L1, and SLC6A1 displayed a more positive association in CRC specimens (Figure 4).

### 3.4. The Expression and Prognostic Value of SLC6A1 in CRC Patients

After screening DNA repair genes, our attention focused on SLC6A1 because its function was rarely reported in CRC. It could be observed that the expression of SLC6A1 was significantly upregulated in CRC specimens than nontumor tissues (Figure 5(a)). Then Kaplan-Meier method suggested that the overall survival of patients with low SLC6A1 expression was better than that of patients with high SLC6A1 expression (*P* = 0.032, Figure 5(b)). More importantly, the multivariate analysis confirmed that the SLC6A1 expression as well as age and clinical stage could be regarded as an independent predicting factor for CRC prognosis (Figures 5(c) and 5(d)).

### 3.5. Functional Enrichment Analysis

According to SLC6A1 mRNA expression, CRC patients in TCGA database were divided into SLC6A1 low expression group and SLC6A1 high expression group, and 42 differentially expressed genes between two groups were screened (Supplementary Table S2). Using the 42 genes, the results of the GO enrichment analysis revealed that the 42 differentially expressed genes were enriched in the extracellular matrix organization, extracellular structure organization, external encapsulating structure organization, collagen-containing, collagen trimer, complex of collagen trimers, extracellular matrix structural constituent, extracellular matrix structural constituent conferring tensile strength, and glycosaminoglycan binding (Figure 6(a)). The KEGG analysis indicated that the differentially expressed genes mainly focused on tumor ECM-receptor interaction, PI3K-Akt signaling pathway, TGF-beta signaling pathway, and proteoglycan (Figure 6(b)).

### 3.6. SLC6A1 Expression Was Negatively Regulated by SLC6A1 Methylation

To explore the mechanisms involved in SLC6A1 dysregulation in CRC, we analyzed the methylation level of SLC6A1 in CRC patients based on TCGA datasets, and the distribution of 13 SLC6A1 CpG sites is clearly shown in Figure 7. The Pearson correlation analysis results showed that the methylation of SLC6A1 DNA methylation, cg11021744, cg23405575, cg19300741, cg07466705, and cg00375819 was negatively correlated with the expression of SLC6A1 (Figures 8(a)–8(f)).

## 4. Discussion

The overall survival rate of patients with CRC has been greatly improved in the field of clinical treatment, but the metastasis and recurrence of CRC are constantly increasing, which is the main cause of CRC death [20, 21]. There is ample evidence that DNA repair genes are a double-edged sword in cancer development [22, 23]. Therefore, new biomarkers based on DNA repair genes are attracting more and more attention.

In this study, we identified 358 abnormally expressed genes between CRC specimens and nontumor specimens and screened 36 survival-related DNA repair genes with a *P* < 0.001. Importantly, we found 10 overlapping DNA repair genes, including ANKLE1, MC1R, TCF7L1, SNAI1, PAXX, WNT3A, TREX2, CDKN2A, SMC1B, and SLC6A1. Some of the above genes have been reported to be dysregulated in several types of tumors and serve as tumor suppressors or promotors [24–28]. Our attention focused on SLC6A1 which was rarely reported in CRC. Previously, Chen et al. reported that SLC6A1 was overexpressed in prostate cancer and its knockdown inhibited the proliferation, migration, and invasion of prostate cancer cells. Besides, its positive association with drug resistance and poor prognosis was also demonstrated in the clinical experiments [29]. This study found that the SLC6A1 expression was significantly elevated in CRC, and the multifactorial analysis showed that the SLC6A1 expression was an independent prognostic marker of the overall survival in CRC patients, which was consistent with the previous findings. In order to further discuss the possible role of SLC6A1 in the CRC progression, we performed KEGG assays with the abnormally expressed genes in CRC specimens with high SLC6A1 expression, and the results revealed that the SLC6A1 expression may be involved in several tumor-related pathways, including PI3K-Akt signaling pathway, relaxin signaling pathway, and TGF-beta signaling pathway. Previous studies have reported that the above three pathways played an important role in the CRC metastasis [30–32]. In addition, several functional genes have been reported to be involved in the CRC progression via modulating the above three pathways [33, 34]. For instance, IMPDH2 promoted the metastasis of CRC cells via regulating the PI3K/AKT/mTOR and PI3K/AKT/FOXO1 signaling pathways [35]. Our findings suggested that SLC6A1 may influence the clinical progression of CRC via modulating the above tumor-related pathways.

The initiation and proliferation of cancer are regulated by epigenetic inheritance and genetic events [36]. Epigenetic modification is increasingly regarded as an important target of cancer research [37]. DNA methylation plays an important role in gene expression and depends on molecular subtypes to influence the prognosis of CRC patients [38, 39]. There is increasing evidence that abnormal DNA methylation plays an important role in the induction and development of CRC [40, 41]. Although many studies have reported the dysregulation of SLC6A1 expression in many types of tumors, its potential mechanisms remained largely unclear [42, 43]. In this study, a strong negative correlation between the SLC6A1 expression and SLC6A1 DNA methylation could be observed. Later, the specific CpG sites were further identified in the SLC6A1 DNA promoter where methylation was significantly associated with SLC6A1 mRNA expression. Unexpectedly, many CpG sites, including cg11021744, cg23405575, cg19300741, cg07466705, and cg00375819, showed significant associations with SLC6A1 expression. Taken together, our findings revealed that SLC6A1 methylation could negatively regulate SLC6A1.

The present study has some limitations. Firstly, the clinical information downloaded from the TCGA databases was limited and incomplete. Secondly, the sample size was relatively small, although the method we developed could eliminate the batch effects. In the future, we will collect more tumor samples to confirm our findings. Moreover, we will also perform in vitro and in vivo experiments to further explore the function of SLC6A1 in the CRC progression.

## 5. Conclusion

To sum up, in this study, the bioinformatics analyses were used to reveal that 36 DNA repair genes were related to cancer progression and prognosis. SLC6A1 was highly expressed in CRC and may serve as a novel prognostic biomarker for CRC patients. Importantly, SLC6A1 was involved in epigenetic modifications, so it may be an outstanding target for cancer therapy.

## Figures and Tables

**Figure 1:** Identification of differentially expressed DNA repair genes in CRC. (a) Volcano plots showed differences in DNA repair gene expression between CRC and nontumor specimens. (b) Hierarchical clustering analysis of differentially expressed DNA repair genes (fold change > 2; *P* < 0.05) in CRC as well as normal tissues.

**Figure 2:** Univariate analysis was used to screen survival-related DNA repair genes in CRC.

**Figure 3:** The identification of dysregulated and survival-related DNA repair genes in CRC. (a) A Venn diagram was used to identify differentially expressed genes associated with overall survival between tumors and adjacent normal tissues. (b) Heat map showed the expression patterns of 10 overlapping genes. (c) Univariate analysis of 10 overlapping genes.

**Figure 4:** Correlation network of the 10 dysregulated and survival-related DNA repair genes in CRC.

**Figure 5:** The expression of SLC6A1 in CRC and its prognostic value. (a) Histogram showed the upregulation of SLC6A1 expression in CRC specimens. (b) Kaplan-Meier plots of SLC6A1 expression in CRC patients. (c) Univariate analysis of SLC6A1. (d) Multivariate analysis of SLC6A1.

**Figure 6:** GO analysis and KEGG pathway analysis of the differentially expressed genes between high SLC6A1 expression group and low SLC6A1 expression group from TCGA datasets. (a) GO enrichment analyses. (b) KEGG pathway enrichment analysis.

**Figure 7:** Histogram of the distribution of 13 SLC6A1 CpG sites in CRC.

**Figure 8:** Correlation analysis of SLC6A1 mRNA expression with DNA methylation. (a) The expression of SLC6A1 was negatively regulated by SLC6A1 DNA methylation. (b–f) Correlation analysis of SLC6A1 mRNA with (b) cg11021744, (c) cg23405575, (d) cg19300741, (e) cg07466705, and (f) cg00375819 methylation.

## Data Availability

The datasets generated during and/or analyzed during the current study are available from the corresponding author on reasonable request.

## Supplementary Materials

Supplementary 1 Table S1: differentially expressed DNA repair genes in CRC specimens from TCGA datasets.

Supplementary 2 Table S2: 42 differentially expressed genes between high SLC6A1 expression and low SLC6A1 group from TCGA datasets.
